RETRACTED

# Establishing an osteosarcoma associated protein-protein interaction network to explore the pathogenesis of osteosarcoma

**DOI:** 10.1186/2047-783X-18-57

**Published:** 2013-12-14

**Authors:** Bi-Yong Deng, Ying-Qi Hua, Zheng-Dong Cai

**Affiliations:** 1 Department of Orthopedic Surgery, Shanghai Tenth people’s Hospital, Tongji University School of Medicine, No.301 Middle Yan-Chang Road, Zha-Bei District, Shanghai 200072, China

**Keywords:** Osteosarcoma, Differentially expressed genes, Protein-protein interaction network, Pathway enrichment analysis

## Abstract

**Background:**

The aim of this study was to establish an osteosarcoma (OS) associated protein-protein interaction network and explore the pathogenesis of osteosarcoma.

**Methods:**

The gene expression profile GSE9508 was downloaded from the Gene Expression Omnibus database, including five samples of non-malignant bone (the control), seven samples for non-metastatic patients (six of which were analyzed in duplicate), and 11 samples for metastatic patients (10 of which were analyzed in duplicate). Differentially expressed genes (DEGs) between osteosarcoma and control samples were identified by packages in R with the threshold of |logFC (fold change)| > 1 and false discovery rate < 0.05. Osprey software was used to construct the interaction network of DEGs, and genes at protein-protein interaction (PPI) nodes with high degrees were identified. The Database for Annotation, Visualization and Integrated Discovery and WebGestalt software were then used to perform functional annotation and pathway enrichment analyses for PPI networks, in which *P* < 0.05 was considered statistically significant.

**Results:**

Compared to the control samples, the expressions of 42 and 341 genes were altered in non-metastatic OS and metastatic OS samples, respectively. A total of 15 significantly enriched functions were obtained with Gene Ontology analysis (*P* < 0.05). The DEGs were classified and significantly enriched in three pathways, including the tricarboxylic acid cycle, lysosome and axon guidance. Genes such as *HRAS*, *IDH3A*, *ATP6ap1*, *ATP6V0D2*, *SEMA3F* and *SEMA3A* were involved in the enriched pathways.

**Conclusions:**

The hub genes from metastatic OS samples are not only bio-markers of OS, but also help to improve therapies for OS.

## Background

Osteosarcoma (OS), an aggressive malignant neoplasm, is the most common primary bone cancer in children and adolescents [1]. Generally, OS occurs in the long bones of the extremities, such as the femur, the tibia and the humerus [2]. Previous studies have demonstrated that it is possible to cure more than 60% of non-metastatic OS with neoadjuvant chemotherapy [3]. However, the 5-year survival rate of patients with metastases at diagnosis is less than 30% [4,5]. Although the mortality has been decreased by about 1.3% per year as a result of improvement in surgical techniques and chemotherapy, there is no reliable means of predicting outcomes at the time of presentation. Thus, identifying potential therapeutic targets is very important in the treatment of patients with metastatic OS.

RETRACTED

OS is a heterogeneous disease including metastatic and non-metastatic complex etiologies. Extensive efforts have been made to explore the underlying pathogenesis and molecular mechanisms. As reported [6], Ezrin links the plasma membrane to the actin cytoskeleton where it plays a pivotal role in the metastatic progression of cancers. Ezrin immunoreactivity can be detected in the majority of patients with non-metastatic OS of the extremity [6]. However, metastatic cells with an efficiently regulated actin cytoskeleton may have a greater fluency and flexibility in managing energetic needs during times of stress than non-metastatic cells. The dysregulation of Ezrin may lead to an urgent but failed attempt by cells to correct this metabolic defect [7]. Therefore, Ezrin is higher expressed in metastatic cells. There are also many other genes that are changed in metastatic OS. *Clusterin*, *collagen 4A3*, *integrin β4*, *integrin β2*, *vascular endothelial growth factor*, *connective tissue growth factor*, *integrin-α5*, *cadherin 2*, *cxc ligand 12*, *cxc chemokin receptor 4*, *cell division cycle 5 like*, and *microRNA215* are found to be upregulated in metastatic OS, while *cadherin 11*, *MME*, *KIAA1959* and *S100A6* are downregulated in metastatic OS [8-11]. Furthermore, some prognosis factors have been demonstrated as potential therapeutic targets, such as reversion-inducing-cysteine-rich protein with kazal motifs and urokinase plasminogen activator [10,11]. The receptor tyrosine kinase-like orphan receptor 2 has also have been identified as being important in the development of metastatic OS [8,12]. In spite of the great progress in the pathogenesis of OS, the molecular mechanisms have not been fully elucidated.

In this paper, we focus on exploring the molecular mechanisms of OS with a computational bioinformatics analysis of gene expression. We anticipate that candidate genes identified by our method may provide a new therapeutic approach for OS.

## Methods

### Affymetrix microarray

The gene profile of GSE9508 was downloaded from the Gene Expression Omnibus (http://www.ncbi.nlm.nih.gov/geo/), which was based on the platform of Agilent-Whole Human Genome Oligo Microarray G4112A, condensed. This expression dataset was deposited by Endo-Munoz [13]. Biopsies were collected at the time of diagnosis, before preoperative chemotherapy, near the tumor-bone interface and were representative of the tumor. A total of 39 samples were derived from 22 patients (11 males and 11 females), including five samples of non-malignant bone (the control), seven samples for non-metastatic patients (six of which were analyzed in duplicate), and 11 samples for metastatic patients (10 of which were analyzed in duplicate). Non-malignant bone was collected from patients presenting for hip or knee replacement surgery.

RETRACTED

### Data processing and identification of differential expression analysis

Firstly, data at the probe-level in CEL format were converted into expression measures and median normalization was performed by R language [14,15]. Then, differentially expressed genes (DEGs) between the samples were identified with the Limma package [16] in R. The Benjamini & Hochberg [17] method was used to adjust the raw *P*-values into the false discovery rate (FDR). |logFC (fold change)| > 1 and FDR < 0.05 were chosen as the cut-off criteria.

### Construction of protein-protein interaction network

The interactions between the DEGs in the groups were analyzed and the protein-protein interaction (PPI) networks were constructed with Osprey using the data from the General Repository for Interaction Datasets [18,19] and Bio-molecular Interaction Network Database [20]. A total of 159 interaction pairs were analyzed.

### Gene ontology enrichment analysis

Gene ontology (GO) analysis has been used frequently in functional studies of large-scale genomic or transcriptomic data [21,22]. GO provides three structured networks of defined terms, namely biological process, molecular function, and cellular compartment [23]. To functionally classify PPI nodes with a high degree (number of interactions), we performed biological process ontology. We performed GO enrichment analysis with The Database for Annotation, Visualization and Integrated Discovery (DAVID), which provides functional interpretation for researchers to study biological information behind large lists of genes [24]. A *P*-value less than 0.05 was considered statistically significant.

### Pathway enrichment analysis

We utilized the WebGestalt web site (web-based gene set analysis toolkit, http://genereg.ornl.gov/webgestalt) [25,26] for pathway enrichment analysis. A *P*-value less than 0.05 was considered as the cut-off criterion.

## Results

### Differential gene expression in osteosarcoma samples

After data normalization (Figure 1), a total of 42 and 341 DEGs with the FDR < 0.05 and |logFC| > 1 were identified between non-metastatic or metastatic samples and the control. These findings indicated that genetic abnormalities in metastatic samples were significantly higher than in non-metastatic samples.

RETRACTED

**Figure 1:** **Normalization of gene expressions in metastatic, non-metastatic and control samples.** The medians (black lines) are almost at the same level, indicating a good level of standardization.

### Protein-protein interaction network

Interaction networks of DEGs were constructed with Osprey (Figure 2A). As a result, interaction relationships of 145 DEGs were obtained. Several PPI nodes were high in degrees in the network, such as POLE (10), HRAS (9), H3F3, HSPA4, ADCY2 (8), IDH3A, ATP6ap1 and ATP6V0D2. All these nodes were obtained from metastatic samples. A high level of connectivity is shown in the network (Figure 2A). All of the five key hub porteins (POLE (10), HRAS (9), H3F3, HSPA4, ADCY2 (8)) and connections were then deleted. As shown in Figure 2B, integrity of the network was disrupted due to the absence of key hubs and connections between the nodes. Compared to the previous network, isolated node clusters were increased in the new network.

**Figure 2:** **Interaction networks of DEGs constructed with Osprey. (A)** Interaction networks of differentially expressed genes constructed with Osprey. **(B)** The integrity of the network was disrupted due to the absence of five key hub proteins (POLE (10), HRAS (9), H3F3, HSPA4, ADCY2 (8)) and connections between the nodes.

### Gene ontology analysis

We performed functional enrichment analysis using the online biological classification tool DAVID, and obtained 15 significantly enriched functions (Table 1, *P* < 0.05). The PPI nodes of high degrees were classified with GO analysis according to their functions. The most remarkable function was regulation of adaptive immune response based on somatic recombination of immune receptors built from immunoglobulin superfamily domains (GO:0002822, *P* = 0.01166). The other significant functions included mRNA metabolic process (GO:0016071, *P* = 0.01427), negative regulation of molecular function (GO:0044092, *P* = 0.02485), nuclear-transcribed mRNA catabolic process (GO:0000184, *P* = 0.02712) and so on. Genes such as *C3*, *TBX21*, *HNRNPL, NCBP2, UPF3A, HRAS, SEMA3F* and *SEM3A* were involved in this GO analysis.

**Table 1:** **Functional enrichment of differentially expressed genes between metastatic samples, non-metastatic samples and non-malignant samples (*P*** **< 0.05)**

**Category**	**Term**	**Count**	***P*-value**	**Genes**
GO:0002822	Regulation of adaptive immune response based on somatic recombination of immune receptors built from immunoglobulin superfamily domains	4	0.01166	*C3, TBX21, RARA, FOXP3*
GO:0002819	Regulation of adaptive immune response	4	0.01225	*C3, TBX21, RARA, FOXP3*
GO:0016071	mRNA metabolic process	9	0.01427	*HNRNPL, NCBP2, UPF3A, C17ORF71, RNMT, GTF2F1, SYNCRIP, SNRPC, SF3A1*
GO:0044092	Negative regulation of molecular function	8	0.02485	*MDFI, KDM1A, ADCY2, RGS3, WWP2, BUB1B, FOXP3, ANGPTL4*
GO:0000184	Nuclear-transcribed mRNA catabolic process, nonsense-mediated decay	3	0.02712	*NCBP2, UPF3A, C17ORF71*
GO:0007626	Locomotory behavior	7	0.03055	*HRAS, CCR3, SEMA3F, MYO15A, CHRNA4, SEMA3A, ESPN*
GO:0051129	Negative regulation of cellular component organization	5	0.03381	*SEMA3F, RDX, CLASP2, SEMA3A, FOXP3*
GO:0048841	Regulation of axon extension involved in axon guidance	2	0.03386	*SEMA3F, SEMA3A*
GO:0048843	Negative regulation of axon extension involved in axon guidance	2	0.03386	*SEMA3F, SEMA3A*
GO:0006370	mRNA capping	2	0.03386	*NCBP2, RNMT*
GO:0000956	Nuclear-transcribed mRNA catabolic process	3	0.03609	*NCBP2, UPF3A, C17ORF71*
GO:0045621	Positive regulation of lymphocyte differentiation	3	0.03609	*RARA, INPP5D, AP3B1*
GO:0051249	Regulation of lymphocyte activation	5	0.03845	*TBX21, RARA, INPP5D, FOXP3, AP3B1*
GO:0009452	RNA capping	2	0.04215	*NCBP2, RNMT*
GO:0050919	Negative chemotaxis	2	0.04215	*SEMA3F, SEMA3A*

RETRACTED

### Pathway enrichment analysis of the protein-protein interaction network

A total of three significant pathways with *P*-value less than 0.05 were enriched (Table 2). The most significant pathway was the citrate cycle (hsa00020, tricarboxylic acid cycle (TCA) cycle) with a *P*-value of 0.006557. Three genes were involved in the TCA cycle, including *SUCLA2, OGDH* and *IDH3A*. The other two significant pathways were the lysosome (*P* = 0.007354) and axon guidance (*P* = 0.009702). Genes associated with the lysosome pathway were *IDS, ATP6AP1, GALNS, ATP6V0D2* and *AP3B1*. Five genes were involved in axon guidance, including *HRAS, RGS3, SEMA3F, SEMA3A*, *APHB1* and *EPHB1*.

**Table 2:** Pathway enrichment in the protein-protein interaction network using the WebGestalt

**Category**	**Count**	***P*-value**	**Differentially expressed genes**
hsa00020: Citrate cycle (TCA cycle)	3	0.006557	*SUCLA2, OGDH, IDH3A*
hsa04142: Lysosome	5	0.007354	*IDS, ATP6AP1, GALNS, ATP6V0D2, AP3B1*
hsa04360: Axon guidance	5	0.009702	*HRAS, RGS3, SEMA3F, SEMA3A, EPHB1*

A total of three significant pathways with *P* < 0.05 were enriched. TCA, tricarboxylic acid cycle.

## Discussion

In the present study, we investigated gene expression profile in OS patients and explored the potential molecular mechanisms using computational bioinformatics methods. Results showed that expressions of 42 and 341 genes were altered in non-metastatic OS and metastatic OS samples, respectively. The DEGs were significantly enriched in three pathways, including the TCA cycle, lysosome and axon guidance. PPI nodes such as HRAS, IDH3A, ATP6ap1 and ATP6V0D2 were of high degrees in the network, all of which were obtained from metastatic samples.

RETRACTED

*IDH3A*, a mitochondrial NAD-dependent isocitrate dehydrogenase involved in the TCA cycle, was identified to exert an effect on OS in our study. OS cells have been demonstrated to have an impaired TCA cycle and partially compensate for the mitochondrial defect [27]. This gene was differentially expressed in metastatic samples compared with the non-metastatic and non-malignant samples, suggesting that *IDH3A* is closely related to migration of metastatic OS cells. In the present study, expression of oncogenic HRAS was increased in metastatic samples. This result was in accordance with a previous study where expression of oncogenic HRAS induced permanent growth arrest in human OS cell lines [28].

Several genes which are specifically found in metastatic OS cells are associated with inhibition of osteoclast differentiation in osteosartic patients, including *ATP6ap1* (Ac45), *ATP6V0D2* (an isoform of V-ATPase subunit d) and *SEMA* (semaphoring). *ATP6ap1*, an accessory subunit of vacuolar-type H + -ATPases (V-ATPases), is identified to be involved in the progress of OS formation. Significantly reduced normal osteoclast formation and inhibition of osteoclast differentiation are found in *Ac45* decreased osteoclast. *Ac45* knockdown leads to the decrease in the number of osteoclasts, which does not result from abnormal apoptosis but from decreased osteoclast precursor cell proliferation and fusion. This decrease is partially due to the downregulation of extracellular signal-regulated kinase phosphorylation and FBJ OS oncogene (c-fos), nuclear factor of activated T-cells, cytoplasmic 1 (NFATc1), and Transmembrane 7 superfamily member 4 expression. Currently, *ATP6ap1* is regarded as a novel therapeutic target for osteolytic disease [29].

*ATP6V0D2* was demonstrated to downregulate the migration of metastatic OS cells in this study. Indeed, it has been identified to mediate osteoclast differentiation [30] and bone formation [31,32]. *ATP6v0d2*, involved in resorption of the bone extracellular matrix, is induced by receptor activator of NF-κB ligand (RANKL) which is necessary for osteoclast formation. Thus, *ATP6v0d2*, as well as *NFAT-c1, TRAP, DC-STAMP* and *cathepsin K*, is considered one of the osteoclast marker genes [33,34].

We also observed the differential expression of semaphoring family genes (*SEMA3F, SEMA3A*), a family of proteins that exert a profound impact on cancers [35]. SEMA3F binds to neuropilin-2 (NRP2) and acts as a tumor suppressor [36]. NRP2 has been reported to affect the increased vascularization and correlate with advanced tumor progression and prognosis in OS [35-38]. Poorer prognosis is related to OS with NRP2 rather than those without NRP2 [38]. In contrast, SEMA-3A binds to NRP1 which induces the collapse of neuronal growth cones. Furthermore, SEMA-3A is induced by RANKL, affecting the osteoblastic profile of OS. This demonstrates that targeting RANK-positive OS may be a novel therapeutic approach [39]. Overall, metastatic cells have been reported more migratory on the premise of bone marrow factors than non-metastatic cells. Furthermore, it is the inherent migratory ability and the sensitivity to osteoclast-mediated inhibition of migration that shows the major differences between metastatic and non-metastatic OS cells [13].

RETRACTED

Although these PPI nodes were isolated and suspected to be involved in the mechanism of metastatic OS, many of them are not shown to participate in this process in experimental research. Further research will be needed to investigate the role played by the genes present in the mechanism of metastatic OS.

## Conclusions

We have demonstrated 42 and 341 DEGs in non-metastatic and metastatic OS samples compared to the control samples. Significantly enriched pathways (including the TCA cycle, lysosome and axon guidance) are dysfunctional in metastatic OS cells. However, the specific markers at the molecular level in the pathogenesis of OS are not fully understood. More studies are warranted to further explore the molecular mechanisms of OS and to apply the molecular genetic diagnosis to the clinic.

## Abbreviations

DAVID: The database for annotation, visualization and integrated discovery; DEG: Differentially expressed gene; FC: Fold change; FDR: False discovery rate; GO: Gene ontology; NFATc1: Nuclear factor of activated T-cells, cytoplasmic 1; NRP2: Neuropilin-2; OS: Osteosarcoma; PPI: Protein-protein interaction; RANKL: Receptor activator of NF-κB ligand; TCA: Tricarboxylic acid cycle.

## Competing interests

The authors declare that they have no competing interests.

## Authors’ contributions

Conceive and design the experiments: ZDC, YQH conceived and designed the experiments. BYD drafted and revised the article, and analyzed and interpreted the data. All authors read and approved the final manuscript.
